The article "Therapeutic interventions impact brain function and promote post-traumatic growth in adults living with post-traumatic stress disorder: A systematic review and meta-analysis of functional magnetic resonance imaging studies" was retracted in 2024. Reasons: unreliable results or conclusions; concerns about the results or conclusions.

# Therapeutic interventions impact brain function and promote post-traumatic growth in adults living with post-traumatic stress disorder: A systematic review and meta-analysis of functional magnetic resonance imaging studies

**DOI:** 10.3389/fpsyg.2023.1074972

**Published:** 2023-02-09

**Authors:** Zachary P. Pierce, Emily R. Johnson, Isabelle A. Kim, Brianna E. Lear, A. Michaela Mast, Jessica M. Black

**Affiliations:** ^1^School of Social Work, Boston College, Chestnut Hill, MA, United States; ^2^The Cell to Society Laboratory, Chestnut Hill, MA, United States; ^3^Department of Neurology, Boston Children's Hospital, Harvard Medical School, Boston, MA, United States

**Keywords:** post-traumatic growth, CPT, EMDR, prolonged exposure, brain, ROI, ALE, meta-analysis

## Abstract

**Introduction:**

The present systematic review and meta-analysis explores the impacts of cognitive processing therapy (CPT), eye movement desensitization and reprocessing (EMDR), and prolonged exposure (PE) therapy on neural activity underlying the phenomenon of post-traumatic growth for adult trauma survivors.

**Methods:**

We utilized the following databases to conduct our systematic search: Boston College Libraries, PubMed, MEDLINE, and PsycINFO. Our initial search yielded 834 studies for initial screening. We implemented seven eligibility criteria to vet articles for full-text review. Twenty-nine studies remained for full-text review after our systematic review process was completed. Studies were subjected to several levels of analysis. First, pre-and post- test post-traumatic growth inventory (PTGI) scores were collected from all studies and analyzed through a forest plot using Hedges’ g. Next, Montreal Neurological Institute (MNI) coordinates and t-scores were collected and analyzed using an Activation Likelihood Estimation (ALE) to measure brain function. T-scores and Hedges’ g values were then analyzed using Pearson correlations to determine if there were any relationships between brain function and post-traumatic growth for each modality. Lastly, all studies were subjected to a bubble plot and Egger’s test to assess risk of publication bias across the review sample.

**Results:**

Forest plot results indicated that all three interventions had a robust effect on PTGI scores. ALE meta-analysis results indicated that EMDR exhibited the largest effect on brain function, with the R thalamus (*t* = 4.23, *p* < 0.001) showing robust activation, followed closely by the R precuneus (*t* = 4.19, *p* < 0.001). Pearson correlation results showed that EMDR demonstrated the strongest correlation between increased brain function and PTGI scores (*r* = 0.910, *p* < 0.001). Qualitative review of the bubble plot indicated no obvious traces of publication bias, which was corroborated by the results of the Egger’s test (*p* = 0.127).

The article "Therapeutic interventions impact brain function and promote post-traumatic growth in adults living with post-traumatic stress disorder: A systematic review and meta-analysis of functional magnetic resonance imaging studies" was retracted in 2024. Reasons: unreliable results or conclusions; concerns about the results or conclusions.

**Discussion:**

Our systematic review and meta-analysis showed that CPT, EMDR, and PE each exhibited a robust effect on PTG impacts across the course of treatment. However, when looking closer at comparative analyses of neural activity (ALE) and PTGI scores (Pearson correlation), EMDR exhibited a more robust effect on PTG impacts and brain function than CPT and PE.

## Introduction

The concept of post-traumatic growth (PTG), devised in the mid-90s by psychologists Tedeschi and Calhoun (1995), describes the process of rebuilding one’s sense of self, others, and the world after experiencing profound (and often chronic) traumatic stress. In contrast to the popular concept of resilience, which refers to the ability of an individual to bounce back when faced with adversity, PTG concerns the *process* of transformation that a survivor undergoes as they move through distress tolerance and narrative reconstruction to incorporate new perspectives about their identities and their relationship to the traumatic event itself (Tedeschi and Calhoun, 2004). This transformative process outlined by PTG has given clinicians, researchers, and survivors a new language with which to describe how to reclaim one’s life from the grips of post-traumatic stress disorder (PTSD).

Current research into PTG has focused primarily on its theoretical construct across clinical contexts (de Sales and Cox, 2004; Pat-Horenczyk and Brom, 2007; Joseph et al., 2012; Jayawickreme et al., 2021) as well as how one might operationalize the psychological components of PTG during experiences of chronic illness (Sherr et al., 2011; Arpawong et al., 2013; Grace et al., 2015; Marziliano et al., 2020; Matos et al., 2021; Yastibas and Karaman, 2021). For example, Grace et al. (2015) explored how individuals can experience PTG after acquired brain injury (ABI) by measuring areas of psychosocial development across the course of treatment. Additionally, Matos et al. (2021) utilized social domains of wellbeing as a measure of PTG for individuals who have experienced COVID-19-related stress. Looking beyond theoretical and psychological constructs, a subset of PTG research within the field of neuroscience has endeavored to identify key brain areas implicated in the phenomenology of PTG.

Wei et al. (2017), for example, have explored how a cohort of adults exposed to the Tianjin explosion incident exhibited greater activation of the left hemisphere of the dorsolateral prefrontal cortex (L dlPFC), which they identify as a crucial region of interest (ROI) implicated in PTG because it regulates distressing affect and irregular heart rate. Similar findings about the L dlPFC were presented by Nakagawa et al. (2016) after assessing survivors of the East Japan Great Earthquake, adding that activation of both hemispheres of the anterior cingulate cortex (L/R ACC) was similarly important because these ROIs help individuals with the synthesis of thoughts and feelings into a self-referential worldview and belief system (Yoshimura et al., 2009; Yang et al., 2012; Nejad et al., 2013; Wagner et al., 2015; Zhao et al., 2018). One might observe that highlighting the L dlPFC over other prefrontal brain regions in the process of PTG may appear odd because it is often the ventromedial prefrontal cortex (vmPFC) that facilitates self-referential cognition in humans (D’Argembeau, 2013; Konu et al., 2020; Park et al., 2020; Stendardi et al., 2021; Yin et al., 2021). With respect to the dlPFC, however, PTG research shows that when compared with other regions in the prefrontal cortex, the dlPFC exhibited the greatest increase in cortical thickness and functional connectivity to other regions (Lyoo et al., 2011; Nakagawa et al., 2016). Why exactly the dlPFC shows greater activity and cortical thickness than the vmPFC during PTG is not outlined in current PTG research. Other studies have identified the L precuneus as a crucial ROI in PTG with respect to its capacity for helping survivors to effectively recode trauma memories and abate the sensitivity of trauma triggers (Stark et al., 2015; Fu et al., 2019). Lastly, various regions across the frontal gyrus have been observed to exhibit significant functions in PTG by restructuring attention to threat stimuli associated with trauma memories as well as thinking creatively about novel ideas and concepts (Hampshire et al., 2010; Japee et al., 2015; Boccia et al., 2015b; Li et al., 2019). Though promising, this subset of PTG research is still in its infancy, affording considerable space for researchers to explore other areas of brain function behind PTG. The same can be said for studies about therapeutic interventions and their impact on PTG brain function (Wagner et al., 2016).

The article "Therapeutic interventions impact brain function and promote post-traumatic growth in adults living with post-traumatic stress disorder: A systematic review and meta-analysis of functional magnetic resonance imaging studies" was retracted in 2024. Reasons: unreliable results or conclusions; concerns about the results or conclusions.

Currently, most studies about PTG brain function during therapeutic treatment have focused on the three leading psychotherapies for PTSD: cognitive processing therapy (CPT), eye movement desensitization and reprocessing (EMDR), and prolonged exposure (PE). To the best of our knowledge, there is yet a study that catalogues findings from all three modalities simultaneously with respect to their correlative impact on PTG and brain function. Thus, we aim to address this gap in the literature with the present systematic review and meta-analysis. Our study will benefit researchers by advancing the knowledge base about the neural bases of PTG across multiple frontline treatments for PTSD. This paper will also bolster the efforts of clinicians by informing them about the effectiveness of psychotherapeutic treatment, promoting the importance of PTG in trauma-informed care, and empowering their clients toward mastering their experiences of trauma survival.

## Methods

### Registration and protocol

Our systematic review and meta-analysis was registered at the International Prospective Register of Systematic Reviews (PROSPERO; ID: CRD42023389058)^1^ and conducted in adherence with the Preferred Reporting Items for Systematic Reviews and Meta-Analyses (PRISMA) guidelines (Page et al., 2021). Our systematic review process was outlined using a PRISMA flow chart (Figure 1). We also utilized the PICOS framework to guide initial construction of our systematic review and meta-analysis protocol. We identified our population and problem area as adults (e.g., individuals ≥18 years old) diagnosed with PTSD. Our identified interventions for this study include CPT, EMDR, and PE. With respect to comparators, our systematic review and meta-analysis provided a comparative analysis between three interventions, and thus a placebo or control group was beyond the scope of this study. Our primary outcome we measured among studies and participants was the prevalence of PTG resulting from treatment. Lastly, the setting in which we conducted this systematic review and meta-analysis was at the Cell to Society Lab at Boston College School of Social Work.

**Figure 1:** PRISMA flow chart of systematic review process.

### Article search and screening process

We utilized four research databases to collect articles for initial assessment before review of eligibility: Boston College Libraries, PubMed, MEDLINE, and PsycINFO. Our search was conducted from March 15, 2022, to March 29, 2022. We collected MeSH terms to serve as the foundation of our keyword search process. Using these terms, we conducted a three-part search process across all databases, utilizing combinations of keywords with increasing specificity for each search. See Figure 2 for an example of our search method and our list of MeSH keywords.

**Figure 2:** Example of systematic search process and keywords.

### Eligibility criteria

We outlined seven criteria by which to include studies for review per precedent established by prior systematic reviews (Henson et al., 2021; Ng et al., 2021):

1. Studies were not systematic reviews and/or meta-analyses.
2. Participants were adults (e.g., individuals ≥18 years old) diagnosed with PTSD according to the *Diagnostic and Statistical Manual of Mental Disorders, Fifth Edition* (DSM-5).
3. Researchers identify CPT, PE, or EMDR as the primary intervention.
4. Studies include pre-and post-treatment post-traumatic growth inventory (PTGI) scores.
5. Researchers utilize concepts germane to PTG (see Figure 2).
6. Studies address brain area function correlated with PTG.
7. Studies include Montreal Neurological Institute coordinates and *t*-scores from functional magnetic resonance imagery (fMRI) procedures.

The article "Therapeutic interventions impact brain function and promote post-traumatic growth in adults living with post-traumatic stress disorder: A systematic review and meta-analysis of functional magnetic resonance imaging studies" was retracted in 2024. Reasons: unreliable results or conclusions; concerns about the results or conclusions.

We included synonyms for PTG in Criterion 5 to control for studies that addressed the phenomenon of PTG but did not use the term directly.

### Interventions

#### Post-traumatic growth inventory

The primary psychometric instrument used to measure PTG across a given intervention in this systematic review and meta-analysis is the Post-Traumatic Growth Inventory (PTGI). Devised by Tedeschi and Calhoun (1996), the PTGI is a 21-item, self-report assessment that measures the cumulative positive psychological changes that occur for a survivor after a traumatic event. The PTGI is often administered in a clinical setting, such as an inpatient or outpatient center. Each item on the PTGI is measured using a 6-point Likert scale, with scores ranging from 0 (“I did not experience this as a result of my crisis”) to 5 (“I experienced this change to a very great degree as a result of my crisis”). Once tabulated each of these items corresponds to one of five factors that create a composite portrait of PTG for a survivor. These factors include (1) personal psychological strength, (2) capacity for envisioning new possibilities, (3) improved social relationships, (4) spiritual (or identity) growth, and (5) appreciation for life. The PTGI has been translated into multiple languages and administered in a variety of cultural contexts, demonstrating high construct validity and reliability in its 10-item short form (Aslam and Kamal, 2019; Garrido-Hernansaiz et al., 2022) as well as its 21-item long form (Gao et al., 2010; Kira et al., 2012; Cadell et al., 2015; Cheng et al., 2017, 2018; Leiva-Bianchi and Araneda, 2015; Mack et al., 2015; Dubuy et al., 2022).

#### Cognitive processing therapy

Cognitive processing therapy (CPT) is a derivative of cognitive behavioral therapy (CBT) that was first devised by Resick and Schnicke (1992) to assist survivors of sexual assault and has since expanded to address traumatic stress in a variety of contexts (Monson et al., 2006; Schulz et al., 2006; Bryant et al., 2011; Galovski et al., 2012; Marques et al., 2016; Ashwick et al., 2019; Bernardi et al., 2019; Galovski et al., 2022). As a 12-session, manualized psychotherapy, CPT guides survivors in a highly organized fashion through the process of addressing traumatic memories as well as targeting and reconstructing beliefs about oneself, others, and the world that undergird these memories (Gallagher and Resick, 2012). CPT invites survivors to reimagine how various domains impacted by traumatic stress have been changed through the course of treatment, such as the client’s sense of power and control, intimacy, safety, self-and other-esteem, and so on. One might observe how internal narrative reconstruction and personal growth throughout the treatment process indicate that CPT has the potential to elicit PTG.

The article "Therapeutic interventions impact brain function and promote post-traumatic growth in adults living with post-traumatic stress disorder: A systematic review and meta-analysis of functional magnetic resonance imaging studies" was retracted in 2024. Reasons: unreliable results or conclusions; concerns about the results or conclusions.

#### Eye movement desensitization and reprocessing

As a progression from traditional exposure therapy paradigms, eye movement desensitization and reprocessing (EMDR) is an intervention that explores how traumatic memories are encoded and how they can be adaptively reorganized to decrease the frequency and intensity of distressing PTSD symptoms (Shapiro, 1989a,b). According to Shapiro (2001), the primary psychological and neural mechanism of change in the phenomenon of traumatic memory reprocessing is bilateral stimulation of the human brain. Both hemispheres are activated either by a client following a clinician’s finger from side to side or utilizing alternating sensory input tools toward the same end, such as pulse paddles, headphones, or foot tapping (Landin-Romero et al., 2018; Hase, 2021). It has been hypothesized that this mechanism of change in EMDR engages ROIs that send cognitions and affects across the corpus callosum, which has been demonstrated to elicit creative thinking about social challenges, cognitive problem solving, and identity reformation, as well as desensitization to and regulation of distressing affects (Wu et al., 2021). Indeed, these functional aspects of EMDR lend themselves toward the possibility of eliciting PTG for survivors undergoing treatment.

#### Prolonged exposure

Prolonged exposure (PE) therapy utilizes a similar cognitive paradigm to CBT but differs insofar that the focus of treatment is on incremental, controlled exposure to a traumatizing stimulus, all with the aim of desensitizing the survivor to threat/fear cues from the stimulus (Foa, 2011). This process of exposure allows individuals to cognitively restructure beliefs about their sense of safety as well as power and control with respect to encountering a traumatizing stimulus in the environment (Hendriks et al., 2018; Rossouw et al., 2018). Typically, PE is structured in 12 90-min sessions and conducted in one of two formats: imaginal exposure or *in vivo* exposure (Foa and Rothbaum, 1998). Imaginal exposure implicates discussion of the trauma stimulus during session where the client creates a verbal/cognitive picture of the stimulus, and then the client revisits this discussion of the stimulus *via* voice recording later on to measure progress in stress response management (Arntz et al., 2007). *In vivo* exposure, on the other hand, implicates clinical “homework” where the client confronts the fear stimulus in a graduated fashion in their social environment outside of therapy (Norr et al., 2019). The psychologically reconstructive components of imaginal and *in vivo* exposure within the framework of PE have the potential to facilitate PTG through rebuilding one’s sense of self and the world by facing a fear stimulus.

The article "Therapeutic interventions impact brain function and promote post-traumatic growth in adults living with post-traumatic stress disorder: A systematic review and meta-analysis of functional magnetic resonance imaging studies" was retracted in 2024. Reasons: unreliable results or conclusions; concerns about the results or conclusions.

### Data extraction

We collected the following items from studies included in our review sample: Author name and year, country where the study took place, sampling type (e.g., convenience or random), total number of participants, mean age and standard deviation of participants, distribution of participant gender identities, context in which the participants’ trauma had taken place (e.g., military service, domestic violence, etc.), intervention type (e.g., CPT, EMDR, or PE), MRI task, T2 and T1 information during fMRI procedures, number of fMRI head channels, coil type, and pre-and post-treatment total PTGI scores with standard deviation. If data were not available in the study, we contacted the authors directly *via* email with request to access data. Data from our review sample were extracted using Microsoft Excel. For data that was not immediately available in the study itself or in supplementary material we contacted authors *via* email for raw data sets.

### Statistical analysis

All statistical analyses were conducted using IBM SPSS 29 and GingerALE Version 3.0.2.^2^ Our primary analysis implicated the effect sizes of PTGI scores between CPT, EMDR, and PE studies. Studies were quantified utilizing *Hedges’ g* with 95% confidence interval (95% CI) based on pre-and post-test PTGI scores and represented in a forest plot (Figure 3). We elected to represent our data using a subgroup analysis to easily trifurcate between CPT, EMDR, and PE groups. This forest plot model also accounted for in-study and between-study variability with *Cochran’s Q*, *Tau*^2^, *H*^2^, and *I*^2^. All studies utilized similar PTGI score procedures and included standard deviation (SD) of scores. Thus, we did not need to make additional considerations during statistical analysis of effect size.

**Figure 3:** Forest plot of PTGI scores.

Next, we conducted a secondary analysis that was divided into two parts. The first part implicated an Activation Likelihood Estimation (ALE) meta-analysis of MNI coordinates and *t*-scores from fMRI procedures across all studies using GingerALE (Table 1; Figure 4). An ALE meta-analysis measures the convergence probabilities of discrete ROIs between experiments, thus seeking to refute the null hypothesis that each experiment impacts ROIs uniformly across the brain (Eickhoff et al., 2012). A standard high-resolution mask was acquired from the Multi-Image Analysis GUI (MANGO)^3^ as a template to house results from our ALE meta-analysis (Figure 4). Table 1 represents quantitative results from images in Figure 4. The second part of our secondary analysis implicated three Pearson correlations, combining data identified in Tables 2, 1. Each Pearson correlation contains results for each modality: CPT (Table 3), EMDR (Table 4), and PE (Table 5).

The article "Therapeutic interventions impact brain function and promote post-traumatic growth in adults living with post-traumatic stress disorder: A systematic review and meta-analysis of functional magnetic resonance imaging studies" was retracted in 2024. Reasons: unreliable results or conclusions; concerns about the results or conclusions.

**Table 1:** Quantitative results from ALE meta-analysis.

Intervention	ROI (Hemisphere)	MNI
		x,y,x	*t*-score	Value of *p*
CPT	STG (R)	−58,60,2	3.29	0.001
	ACC (L)	46,54,-6	3.12	0.002
	Putamen (R)	32,10,-6	4.18	<0.001
	Putamen(L)	−14,10,-6	3.29	0.001
EMDR	Precuneus (L)	6,-60,46	4.19	<0.001
	IFG (L)	46,54,-6	4.12	<0.001
	MFG (R)	−4,54,4	3.27	0.001
	SFG (R)	−20,54,8	2.93	0.003
	IFG (R)	46,54,-6	4.09	<0.001
	Thalamus (R)	20,-9,8	4.23	<0.001
	SFG (L)	−20,54,8	2.30	0.02
PE	Lingual Gyrus (L)	30,-60,4	3.30	0.001
	Insula (R)	40,20,-6	2.82	0.005

Hemisphere: R = right; L = left. ROI: STG = superior temporal gyrus; ACC = anterior cingulate cortex; IFG = inferior frontal gyrus; MFG = middle frontal gyrus; SFG = superior frontal gyrus.

**Figure 4:** Images from ALE meta-analysis. fMR image masks are presented in coronal **(A,B)** and axial **(C,D)** positions. Numeration represents registration of significant ROIs as they appear from quadrant **A** to quadrant **D**. Significant ROIs (and hemispheres): 1. lingual gyrus (L); 2. precuneus (L); 3. STG (L); 4. IFG (L); 5. MFG (R); 6. SFG (R); 7. ACC (L); 8. IFG (R); 9. insula (R); 10. putamen (R); 11. putamen (L); 12. thalamus (R); 13. SFG (L).

**Table 2:** Descriptive statistics from review sample.

Study, year	Context	Sampling	*N*	*M*_age_ [SD]	Gender	Trauma	Int.	MRI	T2		T1		Head	Coil	PTGI scores		(M/F)	Type	Task	TR/TE [ms]	FA	TR/TE [ms]	FA	Pre [SD]	Post [SD]
Aupperle et al., 2013	USA	Convenience	14	40.7 [7.44]	0/14	DV	CPT	FER	2000/32	90°	8/3	8°	32 Ch.	3 T	22.76 [12.18]	88.02 [9.53]
Berman et al., 2018	Israel	Random	68	24.72 [3.89]	0/68	SA	PE	RS	2000/30	75°	25.3/2.88	7°	32 Ch.	3 T	23.82 [15.8]	61.64 [11.01]
Bossini et al., 2012	Europe	Convenience	59	40.8 [13.5]	26/33	DV	EMDR	RS	2000/30	80°	10/4	8°	8 Ch.	1.5 T	25.33 [21.74]	99.46 [15.5]
Bossini et al., 2017	Europe	Convenience	19	40 [9]	10/9	DV	EMDR	RS	9000/110	90°	30/4.6	8°	8 Ch.	1.5 T	25.33 [21.8]	99.48 [15.5]
Boukezzi et al., 2017	Europe	Convenience	18	34.9 [10]	11/7	DV	EMDR	RS	2000/30	80°	9.4/4.42	30°	32 Ch.	3 T	29.83 [8.9]	71.95 [4.27]
Butler et al., 2018	Europe	Convenience	20	27.4 [2.5]	20/0	Military	EMDR	RS	2500/25	80°	22.1/4.7	7°	32 Ch.	3 T	36.88 [7.28]	92.14 [12]
Butler et al., 2020	Europe	Convenience	40	34.2 [7.3]	20/20	Military	EMDR	RS	2500/25	80°	22.1/4.7	7°	32 Ch.	3 T	48.3 [6.3]	91.74 [8.66]
Cisler et al., 2020	USA	Convenience	91	34.5 [8.6]	0/91	CA	PE	RS	2000/30	90°	7.5/3.7	9°	32 Ch.	3 T	55.52 [9.7]	81.5 [11.9]
Etkin et al., 2019	USA	Random	357	40.21 [9.73]	215/142	Military	PE	RS	2000/30	75°	6/3.2	8°	32 Ch.	3 T	43.64 [13.84]	87.47 [10.61]
Fonzo et al., 2017a	USA	Random	66	34.42 [10.23]	26/40	Military	PE	FER	2000/30	80°	8/3.6	15°	8 Ch.	3 T	38.72 [10.61]	73.71 [21.26]
Fonzo et al., 2017b	USA	Random	36	37.72 [9.86]	16/20	Military	PE	FER	2000/30	80°	8/3.6	15°	8 Ch.	3 T	41.56 [11.77]	78.05 [14.5]
Fonzo et al., 2021	USA	Random	66	34.42 [10.23]	26/40	Military	PE	RS	2000/30	80°	8/3.6	15°	8 Ch.	3 T	38.85 [15.17]	87.06 [21.26]
Fujisawa et al., 2015	Asia	Random	33	21.9 [5.7]	12/31	DV	CPT	RS	2300/30	81°	6.38/1.99	11°	32 Ch.	3 T	19.95 [22.2]	91.5 [13.8]
Harlé et al., 2020	USA	Convenience	20	31.95 [7.35]	20/0	Military	PE	RS	2000/32	90°	8/4.8	12°	8 Ch.	3 T	42.06 [15.25]	77.76 [29.08]
Helpman et al., 2016	USA	Random	78	35.9 [9.44]	25/53	DV	PE	FC&E	3000/30	90°	7.25/3	7°	8 Ch.	1.5 T	30.93 [15.6]	78.75 [12.19]
Jung et al., 2016	Asia	Convenience	116	48.44 [6.89]	67/49	Work	PE	RS	2340/35	90°	15/3	15°	8 Ch.	1.5 T	18.38 [15.97]	38.35 [4.69]
Kennis et al., 2015	USA	Convenience	42	33.61 [8.74]	42/0	Military	EMDR	RS	7057/68	90°	66/2.2	18°	32 Ch.	3 T	58.91 [14.37]	73 [15.75]
King et al., 2016	USA	Convenience	19	32.43 [7.54]	10/9	Military	PE	RS	2000/30	90°	9.8/4.6	8°	32 Ch.	3 T	56.71 [18.32]	72.29 [22]
Rousseau et al., 2019a	Europe	Convenience	36	42.25 [7.83]	18/18	DV	EMDR	FER	2530/30	82.4°	9.4/4.42	30°	32 Ch.	3 T	37.3 [18.77]	70.32 [4.49]
Rousseau et al., 2019b	Europe	Convenience	15	36.8 [8.88]	15/0	DV	EMDR	FER	2530/30	82.4°	10/4	30°	32 Ch.	3 T	32.03 [8.13]	81.54 [8.05]
Rousseau et al., 2020	Europe	Convenience	38	32.6 [1.7]	25/13	DV	EMDR	FC&E	2530/30	82.4°	30/3.7	30°	32 Ch.	3 T	30.77 [8.62]	70.55 [7.5]
Santarnecchi et al., 2019	Europe	Random	31	35.4 [14]	18/13	ND	EMDR	RS	2500/32	75°	30/4.6	30°	8 Ch.	1.5 T	30.5 [8.21]	75.6 [11.13]
Simmons et al., 2013	USA	Convenience	31	32.9 [7.2]	31/0	Military	EMDR	PNI	2000/32	90°	8/4	12°	32 Ch.	3 T	25.8 [15.4]	76.7 [16.5]
Thomaes et al., 2016	Europe	Convenience	80	37.4 [8.1]	30/50	SA	EMDR	RS	2000/27.63	76.1°	8.2/3.8	8°	32 Ch.	3 T	25.7 [12.6]	74.8 [24.4]
Van Rooij et al., 2015	Europe	Random	75	34.3 [8.7]	50/25	Military	CPT	G/N-G	1600/23.5	72.5°	10/3.8	8°	32 Ch.	3 T	28.1 [15.2]	94.11 [17.8]
Vuper et al., 2021	USA	Random	42	33.62 [11.1]	0/42	DV	CPT	RS	2200/27	90°	2.4/3.13	8°	32 Ch.	3 T	23.75 [17.71]	87.83 [20.89]
Yang et al., 2018	Asia	Random	104	32.5 [9.72]	10/94	DV	CPT	FER	2000/32	90°	19/3.93	7°	32 Ch.	3 T	21.2 [16.1]	89 [11.6]
Zhu et al., 2018	USA	Convenience	50	35.4 [8.9]	14/36	Military	PE	RS	3000/30	90°	7.25/3	7°	8 Ch.	1.5 T	31.2 [15.2]	72 [22.8]
Zhutovsky et al., 2019	Europe	Convenience	86	33.25 [7.76]	86/0	Military	CPT	RS	1600/23	72.5°	10/4.6	8°	32 Ch.	3 T	29.75 [15.06]	71.92 [16.53]
Total/Mean			1750	35 [7.7]	843/917				2592.8/31.5	81.9°	14.5/3.7	13.3°			33.6 [13.1]	79.6 [14.3]

Trauma Type: DV = domestic violence; SA = sexual assault; CA = child abuse; Work = trauma that occurred as a result of one’s occupation. MRI Task: FER = facial emotion recognition; RS = resting state; FC&E = an unnamed fear conditioning and extinction task; PNI = positive and negative image task; G/N-G = go/no-go impulse task.

The article "Therapeutic interventions impact brain function and promote post-traumatic growth in adults living with post-traumatic stress disorder: A systematic review and meta-analysis of functional magnetic resonance imaging studies" was retracted in 2024. Reasons: unreliable results or conclusions; concerns about the results or conclusions.

**Table 3:** Pearson correlation for brain function and PTG during CPT.

		Brain function	PTGI scores
Brain function	Pearson correlation	1	0.642
	Sig. (2-tailed)		0.170
	N	6	6
PTGI scores	Pearson correlation	0.642	1
	Sig. (2-tailed)	0.170	
	N	6	6

**Table 4:** Pearson correlation for brain function and PTG during EMDR.

		Brain function	PTGI scores
Brain function	Pearson correlation	1	0.910**
	Sig. (2-tailed)		<0.001
	N	12	12
PTGI scores	Pearson correlation	0.910**	1
	Sig. (2-tailed)	<0.001	
	N	12	12

** Correlation is significant at the 0.05 level (2-tailed).

**Table 5:** Pearson correlation for brain function and PTG during PE.

		Brain function	PTGI scores
Brain function	Pearson correlation	1	0.444
	Sig. (2-tailed)		0.171
	N	11	11
PTGI scores	Pearson correlation	0.444	1
	Sig. (2-tailed)	0.171	
	N	11	11

Lastly, we conducted a tertiary analysis to measure risk of bias across all studies (Figure 5). We utilized a bubble plot that measured inverse standard error (ISE) and *Hedges’ g* per the recommendation of Sterne and Egger (2001) and supported by Debray et al. (2018). We elected to include this tertiary analysis because *I^2^* from our forest plot indicated variation in total PANSS scores in and between studies, not publication bias across the studies themselves. Heterogeneity of PTGI scores would not indicate a problem with our meta-analysis because differences in scores served as the primary comparative mechanism for our primary analysis. Our tertiary analysis, therefore, served as a clarifying mechanism for assessing publication bias across all studies.

**Figure 5:** Linear regression of *T*-Scores and *Hedges’ g* values from ALE meta-analysis. Green markers represent coordinates for CPT. Red markers represent coordinates for EMDR. Blue markers represent coordinates for PE.

The article "Therapeutic interventions impact brain function and promote post-traumatic growth in adults living with post-traumatic stress disorder: A systematic review and meta-analysis of functional magnetic resonance imaging studies" was retracted in 2024. Reasons: unreliable results or conclusions; concerns about the results or conclusions.

## Results

### Study selection

Our initial search of all identified databases yielded a total of 834 studies (Figure 1). During initial review 74 duplicate articles were identified and excluded from the initial review pool, and 28 articles were excluded because they were broadly irrelevant to our systematic review and meta-analysis. 732 articles remained for the first stage of screening. The first stage of the screening process subjected articles to two eligibility criteria. The first criterion excluded articles that were systematic reviews and/or meta-analyses (*n* = 116). The second criterion excluded articles where studies did not address adults diagnosed with PTSD (*n* = 6). 610 articles remained for full-text consideration in the second stage of screening. The second stage of screening included five criteria that were used to determine final eligibility in our review sample. Articles were removed that did not include CPT, EMDR, or PE as the primary intervention (*n* = 89), did not include pre-and post-test PTGI scores (*n* = 105), did not include concepts germane to PTG (*n* = 157), did not address brain areas correlated with PTG (*n* = 101), and did not include MNI coordinates and *t*-score data from fMRI procedures (*n* = 129). Twenty-nine studies remained for inclusion in the review sample after this final stage of screening. All studies included relevant data germane to the aims and scope of this systematic review and meta-analysis and did not require further searching or consultation from research teams or associations.

### Study characteristics

Table 2 presents all descriptive statistics collected from articles in our review sample. Contexts for conducting research in our sample featured predominantly in the United States (*n* = 13) and Europe (*n* = 12). Other research contexts included regions of Asia (*n* = 3) and Israel (*n* = 1). With respect to sampling, studies favored a convenience model (*n* = 18) over a random sampling model (*n* = 11). The 29 studies in our sample indicated that 1750 participants were included in all experiments across each modality. The mean age of all participants was 35 years old, with a SD of 7.7 years. Studies featured 917 total female participants and 843 male participants. Studies did not provide information about gender non-binary participants, nor did they include information germane to participant racial or ethnic identities. Contexts for trauma exposure among participants centered around military trauma exposure (*n* = 13) and domestic violence (*n* = 11), which was often characterized by acts of physical aggression between persons. With respect to military trauma exposure, studies did not identify if exposure included military sexual trauma. fMRI tasks among studies frequently utilized a resting state paradigm (*n* = 19) as well a facial emotion recognition tasks (*n* = 6). Others incorporated a positive and negative image task (*n* = 1), a go/no-go task (*n* = 1), and two studies utilized an unnamed fear conditioning and extinction task. T2 weighted imaging processes among studies exhibited a mean TR/TE of 2592.8/31.5 ms with a mean flip angle of 81.9°. T1 weight imaging processes, on the other hand, exhibited a mean TR/TE of 14.5/3.7 ms with a mean flip angle of 13.3°. Most studies in our sample utilized a fMR imaging device with a 32-channel head and 3 Tesla coil magnets (*n* = 19). Lastly, Table 2 includes data of mean pre-and post-test PTGI scores among all participants. The mean pre-test PTGI score among all studies was 33.6, with a SD of 13.1. The mean post-test PTGI scores among all studies was 79.6, with a SD of 14.3.

The article "Therapeutic interventions impact brain function and promote post-traumatic growth in adults living with post-traumatic stress disorder: A systematic review and meta-analysis of functional magnetic resonance imaging studies" was retracted in 2024. Reasons: unreliable results or conclusions; concerns about the results or conclusions.

### Results of individual studies

Our primary analysis included upper and lower 95% CIs and *Hedges’ g* of pre-and post-test PTGI scores in a forest plot (Figure 3). Studies were divided into three subgroups based on treatment modality to compare differences between effect sizes. Following precedent from typical representations of forest plot meta-analyses (Dettori et al., 2021; Chang et al., 2022), we determined that the line of no effect on our forest plot was point 0, where *g* values greater than 0 (or to the right of the line of no effect) indicated that the intervention had a deleterious impact on PTG outcomes. Values less than 0 (or to the left of the line of no effect) indicated that the intervention effectively facilitated PTG. Effects of pre-and post-test PTGI scores for CPT (*g* = −3.93, *p* < 0.001), EMDR (*g* = −3.99, *p* < 0.001), and PE (*g* = −2. 32, *p* = 0.007) were all robust given that they were situated to the left of the line of no effect. Our forest plot included several results for overall heterogeneity: *Tau*^2^ = 2.04; *H*^2^ = 28.35; *I*^2^ = 0.96. It should be noted, however, that these heterogeneity measures—especially *I*^2^—should not be regarded as conclusive. Indeed, in smaller to medium sized meta-analyses *I*^2^ has the potential to overestimate heterogeneity in a review sample by 12–28%, indicating significant bias in the *I^2^* statistic itself (Von Hippel, 2015). Thus, we corrected for this issue by running tests for global homogeneity (*Q* = 451. 13, *df* = 28, *p* < 0.001) and between-subgroup homogeneity (*Q* = 15.9, *df* = 2, *p* < 0.001), both of which indicated marked homogeneity among studies and between subgroups.

The article "Therapeutic interventions impact brain function and promote post-traumatic growth in adults living with post-traumatic stress disorder: A systematic review and meta-analysis of functional magnetic resonance imaging studies" was retracted in 2024. Reasons: unreliable results or conclusions; concerns about the results or conclusions.

Our secondary ALE meta-analysis assessed for frequency of individual ROI activation across all studies using MNI coordinates and *t*-scores (Table 1; Figure 4). Figure 4 is divided into four quadrants, with 4A and 4B offering a coronal view, and 4C and 4D providing an axial view. Each identified ROI is enumerated in the figure legend. Figure 4A indicates primary activation of the L lingual gyrus, L precuneus, and L superior temporal gyrus (STG). Figure 4B indicates primary activation of the L inferior frontal gyrus (IFG), R middle frontal gyrus (MFG), and R superior frontal gyrus (SFG). Figure 4C indicates primary activation of the L ACC, R IFG, R insula, and L/R putamen. Lastly, Figure 4D indicates primary activation of the R thalamus and L SFG. Table 1 shows quantified results from all quadrants of Figure 4 to assess which ROIs were activated during each intervention and determine how significant these activations were in comparison to other identified ROIs. Results from Table 1 indicated that EMDR exhibited the strongest prevalence of ROI activation across all modalities (L precuneus: *t* = 4.19, *p* < 0.001; L IFG: *t* = 4.12, *p* <. 001; R MFG: *t* = 3.27, *p* = 0.001; R SFG: *t* = 2.93, *p* = 0.003; R IFG: *t* = 4.09, *p* < 0.001; R thalamus: *t* = 4.23, *p* < 0.001; L SFG: *t* = 2.30, *p* = 0.02). Table 1 also showed some significant ROI activation during CPT (R STG: *t* = 3.29, *p* = 0.001; L ACC: *t* = 3.12, *p* = 0.002; R putamen: *t* = 4.18, *p* < 0.001; L putamen: *t* = 3.29, *p* = 0.001) and PE (L lingual gyrus: *t* = 3.30, *p* = 0.001; R insula: *t* = 2.82, *p* = 0.005).

### Synthesis of results

We elected to synthesize results from our primary and secondary analyses using the conventional method of the Pearson correlation (Cohen and Kohn, 2011). We conducted three Pearson correlations in total: one for CPT (Table 3), EMDR (Table 4), and PE (Table 5). Each Pearson correlation utilized *Hedges’ g* values from our forest plot (representing effect for PTGI scores) and *t*-scores from our ALE meta-analysis (representing effect for brain function). Our primary objective with these Pearson correlations was to assess if there was a positive correlation between brain function and PTGI scores: i.e., Does one’s brain function during treatment positively correlate with an increase in PTG? Table 3 indicates that CPT had a moderate positive correlation between brain function and PTGI scores (*r* = 0.642, *p* = 0.170). Table 5 offers a similar result for PE (*r* = 0.444, *p* = 0.171). Table 4, however, demonstrates that EMDR exhibited a robust positive correlation between brain function and PTGI scores (*r* = 0.910, *p* < 0.001). For reader convenience we have included a linear regression of *Hedges’ g* values and *t*-scores from our ALE meta-analysis to directly compare outcomes from our Pearson correlations (Figure 5).

The article "Therapeutic interventions impact brain function and promote post-traumatic growth in adults living with post-traumatic stress disorder: A systematic review and meta-analysis of functional magnetic resonance imaging studies" was retracted in 2024. Reasons: unreliable results or conclusions; concerns about the results or conclusions.

### Risk of bias across studies

To conclude statistical analyses conducted in our systematic review and meta-analysis, we utilized a bubble plot to assess risk of bias across studies in our review sample. We utilized a bubble plot with Egger’s test of random effects to avoid the risks of bias presented by *I*^2^ mentioned above. Upon qualitative review, Figure 6 presents a generally symmetrical distribution of studies along the axes of inverse standard error and *Hedges’ g*. Our review was corroborated by intercept results of the Egger’s test, which indicated that our risk of bias through heterogeneity and lack of precision across studies was statistically insignificant (*p* = 0.127).

**Figure 6:** Bubble plot of risk of bias across studies. Egger’s test: *p* = .127.

## Discussion

The present systematic review and meta-analysis aimed to assess the relationship between brain function and PTG among three gold standard psychotherapeutic interventions for PTSD: CPT, EMDR, and PE. Results from our forest plot indicated that all three interventions had a profound effect on PTGI scores across treatment. In particular, EMDR (*g* = −3.99, *p* < 0.001) and CPT (*g* = −3.93, *p* < 0.001) exhibited similarly robust effects on PTGI scores across treatment followed by PE (*g* = −2.32, *p* = 0.007). Based on the role of the PTGI as a psychometric instrument for effectively measuring PTG, we infer from our findings indicate that all three interventions can effectively facilitate PTG for individuals undergoing treatment, which is an encouraging prospect for trauma clinicians a researchers alike.

With respect to brain function, our ALE meta-analysis presented some interesting findings with respect to each intervention as well as known ROI activity during PTG. Figure 4 and Table 1 demonstrated that EMDR had a more pronounced impact on estimated ROI activation during treatment when compared with CPT and PE. Activation of the superior, middle, and inferior regions of the frontal gyrus are unsurprising in EMDR given that these areas are principally implicated in the psychological processes of creative problem solving and belief reconstruction vis-á-vis bi-hemispherical stimulation (Pagani et al., 2015; Boccia et al., 2015a). It is also noteworthy that these psychological processes of EMDR are also crucial elements of the process of PTG (Boccia et al., 2015b). Though tangentially related, one might also say the same about the activation of the R thalamus. The R thalamus is principally responsible for relaying afferent sensory stimuli from the autonomic nervous system (ANS) to the frontal lobe for further cognitive processing (Wolff and Vann, 2019; Pierce and Black, 2021). When one considers the frequency and intensity of distressing ANS stimuli that one might experience during acute PTSD symptoms (e.g., racing heart, shortness of breath, muscle tension, increased sweat secretion, etc.), the increased regulatory capacity of the thalamus is paramount toward curating an internal sense of safety for a survivor, without which the process of PTG might be thwarted (Zhou et al., 2019; Kapur et al., 2022). Lastly, the L precuneus, among its many functions, is often implicated in novel environmental information processing and integration as well as stressful cue reactivity inhibition (Geuze et al., 2007; Sartory et al., 2013). When filtered through the psychological lens of PTG, these two functions of the L precuneus aid survivors in restructuring one’s internal narrative based on novel information and promoting the extinction of a fear response to a traumatizing stimulus—a small but no less important part of PTG (Norrholm et al., 2011; Zuj et al., 2016).

The article "Therapeutic interventions impact brain function and promote post-traumatic growth in adults living with post-traumatic stress disorder: A systematic review and meta-analysis of functional magnetic resonance imaging studies" was retracted in 2024. Reasons: unreliable results or conclusions; concerns about the results or conclusions.

Increased activation of the L ACC during CPT is expected given that a central component of this intervention implicates exercises that challenge and restructure beliefs about oneself, others, and the world related to the traumatic event. It is also unsurprising to find that both hemispheres of the putamen are activated during CPT. Both L/R putamen are implicated in cognitive processing of language and spoken language articulation (Viñas-Guasch and Wu, 2017). During CPT the client is invited to write out two impact statements (one at the beginning and end of treatment) and multiple detailed trauma accounts. Each of these statements and accounts are read aloud multiple times during different sessions by the client. As these literary items are read by the client, the clinician encourages the client to notice changes in how they read certain sentences or phrases as well as when they encounter a ‘stuck point’, i.e., a place in the narrative that is affectively painful to recount or difficult to remember. All these elements of the therapeutic process of CPT are correlated with the functions of the putamen. We also observe how these elements of CPT play a role in the activation of the R STG, which is responsible for auditory processing of lingual and sonic stimuli (Hullett et al., 2016). Reading one’s impact statement or trauma account aloud multiple times and thinking critically about various parts of these literary items certainly recruits the STG to assist in processing one’s speech. We suggest that these roles of the L/R putamen and R STG are tangential to the process of PTG. For example, these ROIs contribute to the efforts of the L ACC to assist in restructuring one’s beliefs by processing how these beliefs change across trauma accounts and impact statements.

The article "Therapeutic interventions impact brain function and promote post-traumatic growth in adults living with post-traumatic stress disorder: A systematic review and meta-analysis of functional magnetic resonance imaging studies" was retracted in 2024. Reasons: unreliable results or conclusions; concerns about the results or conclusions.

With respect to PE, we expected that increased activity of the insula would figure with some prominence among other ROIs during this intervention. Indeed, the R insula is responsible for emotion regulation and the extinction of pain and fear responses to distressing environmental stimuli (Uddin et al., 2017). Given that PE clinicians invite clients to master traumatizing events by incrementally exposing themselves to the stimulus, increased activity and regulation *via* the R insula coheres with the therapeutic ends of PE. However, we did not expect prominent activation of the L lingual gyrus during PE. We hypothesize that significance of the L lingual gyrus is derived from two functions. First, the L lingual gyrus has been observed to be a mediating factor for divergent thinking (i.e., racing thoughts) during episodes of anxiety (Zhang et al., 2016). As has been discussed, this function serves an ancillary role for helping survivors feel safe enough to explore the process of PTG. Second, the L lingual gyrus has been shown to function as an important node of connection between the limbic system, default mode network, and salience network, aiding in the process of declarative memory reconstruction and emotion processing in resilient individuals after experiencing childhood PTSD (Van der Werff et al., 2013). To what end the lingual gyrus is directly implicated in these processes is unknown. However, its relationship to these processes can be determined to be, likewise, tangential.

Our results are surprising, broadly speaking, because nowhere did activation of the dlPFC feature. As was discussed in the introduction to this systematic review and meta-analysis, previous studies had identified the dlPFC as a prominent ROI in the process of PTG because its functions help to facilitate this process (Nakagawa et al., 2016; Wei et al., 2017). We are unsure why the dlPFC did not figure in our ALE meta-analysis. However, we have two hypotheses: (1) The function of the dlPFC is not as important to the process of PTG as was once thought, or (2) more studies are needed to flesh out the role of the dlPFC in the process of PTG.

Lastly, to explore the nuance between large effect scores in our forest plot and determine if there was a relationship between brain function and PTG, we synthesized data from Table 1 and Figure 3 using Pearson correlations (see also Figure 5). Data representing brain function implicated *t*-scores from frequently activated ROIs in Table 1. Data representing PTG implicated PTGI score effect sizes *via Hedges’ g* values from Table 3. Tables 3, 5 indicated that CPT (*r* = 0.642, *p* = 0.170) and PE (*r* = 0.444, *p* = 0.171) each exhibited moderate positive correlations between brain function and PTGI scores. Minute differences between these correlations become apparent in Figure 5 where the line of best fit for PE coefficients (colored blue) shows a slight increase of neural activity as PTGI scores increase, and the line of best fit for CPT coefficients (colored green) exhibits a more pronounced increase in neural activity as PTGI increases. Table 4, however, shows that EMDR exhibited a robust positive correlation between brain function and PTGI scores (*r* = 0.910, *p* < 0.001). The magnitude of this correlation is indicated by EMDR coefficients (colored red) closely matching with the line of best fit when compared with CPT and PE coefficients (Figure 5). Thus, we infer from our Pearson correlation findings that EMDR exhibits a stronger impact than CPT and PE on promoting ROI activation and facilitating PTG.

The article "Therapeutic interventions impact brain function and promote post-traumatic growth in adults living with post-traumatic stress disorder: A systematic review and meta-analysis of functional magnetic resonance imaging studies" was retracted in 2024. Reasons: unreliable results or conclusions; concerns about the results or conclusions.

## Limitations

Though our systematic review and meta-analysis offers important findings regarding the psychotherapeutic relationship between brain function and PTG, several limitations exist. First, we recognize that studies were conducted across different sites, using different fMRI tasks, and that these variables have the potential to impact which ROIs might activate during treatment. Thus, when describing the neural phenomenology of PTG, it is imperative to note these factors as they can change the discussion of which ROIs might activate during this psychological process and why they do so. This limitation does not, however, impact findings presented in this systematic review and meta-analysis because, given the limitations of available studies, we created to the best of our ability a portrait of brain function that occurs during PTG across these disparate settings. To add clarity to the neural processes implicated in PTG, we encourage future studies to utilize similar sites and protocol to control for these discrepancies. Participants in our review sample encompass a limited demographic range. While our systematic review and meta-analysis offers a broad view about neural correlates associated with PTG among CPT, EMDR, and PE, the nuances of gender and racial identity and their impacts on brain function were not captured due to not being included in surveyed studies. For example, it is unclear if individuals who identify as non-binary participated in studies included in our review sample because these data were not featured. Historically marginalized populations, such as BIPOC individuals, were under-reported among study samples, limiting the discussion about how trauma might uniquely impact these populations.

The article "Therapeutic interventions impact brain function and promote post-traumatic growth in adults living with post-traumatic stress disorder: A systematic review and meta-analysis of functional magnetic resonance imaging studies" was retracted in 2024. Reasons: unreliable results or conclusions; concerns about the results or conclusions.

Next, we recognize that while our bubble plot sufficiently assesses risk of bias across our review sample, our systematic review and meta-analysis would have further benefited from the inclusion of the QUADAS-2 instrument to assess individual article quality. The QUADAS-2 instrument measures individual risk of bias across four domains: patient selection, index testing, reference standard, and flow and timing (Whiting et al., 2011). We encourage future systematic reviews and meta-analyses to incorporate this instrument to bolster findings about risk of bias within review samples.

Additionally, our ALE meta-analysis was unable to capture the temporality of activation between individual ROIs in our review sample. With respect to Figure 4B, for example, we are unable to determine if the L IFG activated before, after, or concurrently with the R MFG and SFG during EMDR. We were able to make general inferences about patterns of activation of these ROIs based on the therapeutic mechanisms of EMDR, but we could not determine the specific timing of ROI activation based on the data alone. More research is needed to determine temporal aspects of ROI activation during psychotherapeutic treatment.

Lastly, MNI coordinates and *t*-scores from fMRI data were obtained shortly after graduation from each treatment and does not describe long-term brain function and PTG. Further research is needed to determine the long-term efficacy of each intervention toward sustaining PTG and its concomitant impacts on brain function.

## Future directions

Based on findings from our systematic review and meta-analysis, we recommend several avenues for future research, practice, and policy development and advocacy. First, systematic reviews and/or meta-analyses of longitudinal studies exploring the impact of PTSD treatment on ROI activity over time and in the context of remission or relapse would offer a more comprehensive view of PTG neuroanatomy. Another area for exploration not incorporated in this analysis is the impact of PTSD treatment on neural development in children and youth and the impact of possible epigenetics and historical trauma on baseline PTG ROI functioning that may impact predisposition or resilience to developing PTSD as well as the impact of PTSD treatment for these individuals. Further research may also examine more thoroughly how ROI activity might be associated with protective and risk factors associated with PTG.

The article "Therapeutic interventions impact brain function and promote post-traumatic growth in adults living with post-traumatic stress disorder: A systematic review and meta-analysis of functional magnetic resonance imaging studies" was retracted in 2024. Reasons: unreliable results or conclusions; concerns about the results or conclusions.

Within the scope of mental healthcare practice, clinicians who specialize in trauma-informed care might utilize our data to promote effective psychoeducation for survivors about the brain function behind their experience of PTSD symptoms and the phenomenon of PTG. As the neuroscientific community continues to expand its knowledge base about the foundation of neural activity implicated in trauma survival, this knowledge can continue to be translated as has been done here for consumption by clinicians. Not only would our data enhance the expertise of clinicians delivering services but also equip survivors with knowledge about their bodies, affording them renewed access to a sense of control over the tumult of trauma survival. These data might also encourage clinicians to explore training in frontline treatments for PTSD, such as EMDR, CPT, and PE. Combining practice knowledge from these interventions in the field with insights from our systematic review and meta-analysis would help clinicians gain a holistic perspective of trauma treatment, addressing specific elements of human psychology and brain function implicated in PTG toward one’s comprehensive goals in trauma treatment.

Lastly, we encourage increased efforts in policy development and advocacy across two domains. The first domain implicates increased access to translated neuroscientific data for public consumption, especially with respect to the impact of PTG on the human brain. Allowing a wider array of access to these kinds of insights would allow more individuals to learn about the biological underpinnings of trauma survival and growth and how they might address these areas during treatment. A policy of this scope would be particularly relevant for individuals from historically marginalized communities, as these populations often experience a greater frequency of traumatic events, yet do not have access to scientific resources that might aid in their survival and their progression through PTG. The second domain includes greater access to affordable training for trauma-informed interventions. As is often the case, trainings for therapeutic treatment delivery are obfuscated behind paywalls that are too high for the average clinician to surmount (Crome et al., 2017). It is also the case that the average clinician does not receive institutional support toward paying for these trainings (Okamura et al., 2018). EMDR, CPT, and PE are no exception. Presenting trainings for these interventions more frequently and at an affordable rate would allow more trauma survivors to receive an adequate level of care. Most importantly, increasing the availability of these interventions would present survivors with hope—a chance to experience positive change and growth after what surely has felt like a lifetime of hellacious, all-consuming overwhelm.

The article "Therapeutic interventions impact brain function and promote post-traumatic growth in adults living with post-traumatic stress disorder: A systematic review and meta-analysis of functional magnetic resonance imaging studies" was retracted in 2024. Reasons: unreliable results or conclusions; concerns about the results or conclusions.

## Data availability statement

The original contributions presented in the study are included in the article/supplementary material, further inquiries can be directed to the corresponding author.

## Author contributions

All authors contributed equally in the conceptualization, research, drafting, and completion of this manuscript. All authors contributed to the article and approved the submitted version.

## Conflict of interest

The authors declare that the research was conducted in the absence of any commercial or financial relationships that could be construed as a potential conflict of interest.

## Publisher’s note

All claims expressed in this article are solely those of the authors and do not necessarily represent those of their affiliated organizations, or those of the publisher, the editors and the reviewers. Any product that may be evaluated in this article, or claim that may be made by its manufacturer, is not guaranteed or endorsed by the publisher.

## Footnotes

^1^ https://www.crd.york.ac.uk/PROSPERO

^2^ https://brainmap.org/ale/

^3^ https://mangoviewer.com/
